The article "Prognosis and Efficacy of Laparoscopic Surgery on Patients with Endometrial Carcinoma: Systematic Evaluation and Meta-Analysis" was published in 2022. Journal: Comput Math Methods Med.

# Prognosis and Efficacy of Laparoscopic Surgery on Patients with Endometrial Carcinoma: Systematic Evaluation and Meta-Analysis

**DOI:** 10.1155/2022/9384134

**Published:** 2022-09-22

**Authors:** Jiong Ma, Chunxia Zhou, Jinyan Chen, Xuejun Chen

**Affiliations:** Department of Gynecology, Second Affiliated Hospital, Zhejiang University, School of Medicine, Hangzhou, Zhejiang 310009, China

## Abstract

**Objective:**

The prognosis and efficacy of laparoscopic surgery (LPS) and open surgery or robotic surgery (RS) on endometrial carcinoma (EC) patients were compared.

**Methods:**

Data as of May 2021 were retrieved from databases like PubMed, Embase, Cochrane Library, and Web of Science. The study involved randomized controlled trials (RCTs), cohort studies, or case-control studies for comparing the effects of LPS and open surgery or robotic surgery (RS) on EC treatment. The primary outcomes included duration of operation, blood loss, length of stay (LOS), postoperative complications, and recurrence rate. Secondary outcomes included 3-year progression-free survival (PFS) rate/disease-free survival (DFS) rate and 3-year overall survival (OS) rate.

**Results:**

A total of 24 studies were involved, and all of them were cohort studies except 1 RCT and 1 case-control study. There was no significant difference in duration of operation between LPS and open surgery (MD = −0.06, 95% CI: -0.37 to 0.25) or RS (MD = −0.15, 95% CI: -1.27 to 0.96). In comparison with the open surgery, LPS remarkably reduced blood loss (MD = −0.43, 95% CI: -0.58 to -0.29), LOS (MD = −0.71, 95% CI: -0.92 to -0.50), and the complication occurrence rate (RR = 0.83, 95% CI: 0.73 to 0.95). However, LPS and RS saw no difference in blood loss (MD = 0.01, 95% CI: -0.77 to 0.79). Besides, in comparison with RS, LPS prominently shortened the LOS (MD = 0.26, 95% CI: 0.12 to 0.40) but increased the complication occurrence rate (RR = 1.74, 95% CI: 1.57 to 1.92). In contrast to open surgery or RS, LPS saw no difference in occurrence rate (RR = 0.75, 95% CI: 0.56 to 1.01; RR = 0.97, 95% CI: 0.62 to 1.53), 3-year PFS/DFS (RR = 0.99, 95% CI: 0.90 to 1.09; RR = 1.30, 95% CI: 0.87 to 1.96), and 3-year OS (RR = 0.97, 95% CI: 0.91 to 1.04; RR = 1.21, 95% CI: 0.91 to 1.60).

**Conclusion:**

In sum, LPS was better than open surgery, which manifested in the aspects of less blood loss, shorter LOS, and fewer complications. LPS, therefore, was the most suitable option for EC patients. Nevertheless, LPS had no advantage over RS, and sufficient prospective RCTs are needed to further confirm its strengths.

## 1. Introduction

Endometrial carcinoma (EC) is the most commonly diagnosed gynecologic malignant tumor, especially in some developed countries [1], whose 5-year survival rate was 34.7% (445805 cases) [2]. The risk factors of EC include early menarche, delay menopause, diabetes, polycystic ovarian syndrome (PCOS), metabolic syndrome, current treatments with tamoxifen, and obesity [3–5]. With the increase of risk factors such as aging of population and obesity, the morbidity of EC will continue to rise. Most EC patients who are diagnosed in the early stages (Federation Internationale of Gynecologie and Obstetrigue (FIGO) stage I or II) have better prognoses [6].

The article "Prognosis and Efficacy of Laparoscopic Surgery on Patients with Endometrial Carcinoma: Systematic Evaluation and Meta-Analysis" was published in 2022. Journal: Comput Math Methods Med.

Surgeries remain the major treatment for early EC, which mainly include vaginal surgery, laparotomy (LT), or open surgery, laparoscopic surgery (LPS), and robotic surgery (RS). Clinical practice guideline and multiple clinical trials indicate that minimally invasive surgery (MIS) is recommended as the preferred surgical approach for EC patients [7, 8]. In the past, LT has always been the first choice for early EC patients. Since the first report of LPS on EC in 1993 [9], LPS, as a MIS, has become increasingly popular in the treatment of EC [10, 11]. In contrast to open surgery, LPS is characterized by less blood loss, less renascent adhesion and lower morbidity [12]. RS is a new MIS developed on the basis of LPS. Previous studies show that RS for EC treatment results in a shorter length of stay (LOS), less blood loss, lower conversion rate of open surgery, and lower occurrence rate of intraoperative damage to surrounding organs, compared to LPS [13, 14]. However, in contrast to LPS, RS prolongs operation and recovery time [15, 16]. Recently, a multicenter retrospective study compared the therapeutic efficacy of LPS and radical abdominal hysterectomy on early EC patients. The result indicated a decrease in the disease-free survival (DFS) of patients who underwent LPS [17]. However, a prospective study validated that LPS could dramatically improve the short- and long-term quality of life (QOL) of EC patients [18]. Hence, this study systematically evaluated the prognosis and efficacy of LPS.

Consequently, we conducted a meta-analysis to elucidate the prognosis and effect of LPS on EC by comparison with open surgery or RS from the perspective of perioperative results, postoperative complications, recurrence rate, and survival time. This effort will bring insight into the surgical treatment of EC patients.

## 2. Methods

### 2.1. Literature Retrieval

The study was performed in adherence to the Preferred Reporting Items for Systematic reviews and Meta-Analyses (PRISMA) statement [19]. All relevant literature included in the databases like PubMed, Embase, Cochrane Library, and Web of Science were retrieved from the construction of the databases to May 2021. Keywords used for searching included “endometrial carcinoma,” “hysteroscopic surgery,” “minimally invasive surgery,” “laparoscopic surgery,” “robotic surgery,” and “open surgery.” The detailed strategy of literature retrieval was as follows: ((((Endometrial Neoplasm^∗^[MeSH Terms]) OR (Endometrial Carcinoma^∗^[MeSH Terms])) OR (Endometrial Cancer^∗^[MeSH Terms])) AND (((((Laparoscopy[Title/Abstract]) OR (Hysteroscope[Title/Abstract])) OR (Minimally invasive[Title/Abstract])) OR (Open[Title/Abstract])) OR (robotic[Title/Abstract]))) AND ((operation[Title/Abstract]) OR (surgery[Title/Abstract])).

The article "Prognosis and Efficacy of Laparoscopic Surgery on Patients with Endometrial Carcinoma: Systematic Evaluation and Meta-Analysis" was published in 2022. Journal: Comput Math Methods Med.

### 2.2. Selection of Studies

Inclusion criteria of the literature were as follows: (1) patients diagnosed with EC; (2) comparison between effects of LPS and open surgery or RS on EC treatment; (3) at least one of the results such as duration of operation, blood loss, LOS, postoperative complications, recurrence rate, 3-year progression-free survival (PFS) rate/DFS rate, and 3-year overall survival (OS) rate was reported; and (4) study was designed as RCT, cohort study, or case-control study. The following were the exclusion criteria of the literature: (1) repeated publication, case series, case report, comments, meeting abstract, review, editorial, letter, and so on; (2) data were not sufficient to obtain the result of our study; (3) article replications; and (4) studies lack of efficacy-related data.

### 2.3. Data Extraction and Quality Assessment

The information obtained from the literature included the information of the authors, publication year, country, study design, the year the samples were collected, the number of samples, and intervening measures. Data of the patients included age, body mass index (BMI), FIGO stage, pathological grading, and outcome indicator. Primary outcomes included duration of operation, blood loss, LOS, and postoperative complications. Secondary outcomes involved postoperative recurrence rate, 3-year PFS rate/DFS rate, and 3-year OS rate.

Cochrane risk of bias assessment tool was employed to assess the quality of RCT which was graded as “low risk,” “high risk,” and “uncertain risk.” Besides, the Newcastle-Ottawa Scale (NOS) was utilized to evaluate the risk of publication bias in observational studies. Aggregate points of NOS were 9, and literature with the points greater than or equal to 6 was considered of good quality.

The search and selection of articles and the extraction and quality evaluation of data were independently finished by two investigators. Disputes were solved by the third investigator through consultation.

### 2.4. Statistical Analysis

Meta-analysis was performed using the Stata 16.0 software. Continuous data were expressed as mean ± standard deviation (SD). Mean difference (MD) was measured via continuous results, and 95% confidence intervals (CIs) were used to assess the concrete therapeutic effect. If CI included 0, it denoted no statistical difference between two groups. Besides, two-category data were merged and analyzed utilizing relative risk (RR) and their 95% CI. If CI included 1, it indicated no statistical difference between two groups. *I*^2^ statistic was applied to assess the statistical heterogeneity of studies involved. A random effect model was used if *p* < 0.1 or *I*^2^ > 50%, suggesting a remarkable heterogeneity. Otherwise, a fixed effect model was used.

The article "Prognosis and Efficacy of Laparoscopic Surgery on Patients with Endometrial Carcinoma: Systematic Evaluation and Meta-Analysis" was published in 2022. Journal: Comput Math Methods Med.

## 3. Results

### 3.1. Screening and Selection of Reports

A total of 1666 reports were retrieved based on the established searching strategies, among which 224 reports were excluded. Further, 1400 reports were excluded by scanning their title and abstract. After reading the full text of the remaining 42 reports, 7 reports of them reported unrelated data while 11 of them lacked sufficient data for obtaining the result of our study. Finally, 24 reports were selected for our study [13, 20–42]. The procedures of report screening are shown in Figure 1.

### 3.2. Characteristics of the Studies and Quality Evaluation

A total of 24 reports were involved in the study, in which 6814 patients underwent LPS and 5315 patients underwent open surgery. Besides, 6121 patients underwent RS. Except for 1 RCT and 1 case-control study, the other reports were cohort studies. All characteristics of reports involved and the results of quality assessment are displayed in Table 1. Papers with the points greater than or equal to 6 were of high quality.

### 3.3. Results of Meta-Analysis

#### 3.3.1. Duration of Operation and Blood Loss

In respect of the operation time, 9 studies compared that in LPS and open surgery (*I*^2^ = 95.2%), and 2 studies compared that in LPS and RS (*I*^2^ = 98.0%). Due to huge heterogeneity, a random effect model was introduced for analysis. The outcome of meta-analysis suggested that there was no significant difference in duration of operation between LPS and open surgery (MD = −0.06, 95% CI: -0.37 to 0.25) or RS (MD = −0.15, 95% CI: -1.27 to 0.96) (Figures 2(a) and 2(b)).

In respect of blood loss, 6 studies compared that in LPS and open surgery (*I*^2^ = 47.1%), and 2 studies compared that in LPS and RS (*I*^2^ = 96.0%). Based on the results of heterogeneity analysis, a fixed effect model and a random effect model were employed, respectively. The result of meta-analysis demonstrated that the blood loss of LPS was dramatically decreased in contrast to open surgery (MD = −0.43, 95% CI: -0.58 to -0.29), but it had no remarkable difference when compared with that of RS (MD = 0.01, 95% CI: -0.77 to 0.79) (Figures 3(a) and 3(b)).

The article "Prognosis and Efficacy of Laparoscopic Surgery on Patients with Endometrial Carcinoma: Systematic Evaluation and Meta-Analysis" was published in 2022. Journal: Comput Math Methods Med.

#### 3.3.2. Postoperative LOS, Complications, and Recurrence Rate

In respect of LOS, 5 studies compared that in LPS and open surgery (*I*^2^ = 72.1%), and 2 studies compared that in LPS and RS (*I*^2^ = 0.0%). Based on the results of heterogeneity analysis, a random effect model and a fixed effect model were employed, respectively. It was exhibited in meta-analysis that the LOS of LPS was shorter than that of open surgery (MD = −0.71, 95% CI: -0.92 to -0.50) (Figure 4(a)). Meanwhile, the LOS of RS was shorter by comparison with that of LPS (Figure 4(b)).

In respect of postoperative complications, 15 studies compared that in LPS and open surgery (*I*^2^ = 83.3%), and 8 studies compared that in LPS and RS (*I*^2^ = 76.6%). Due to huge heterogeneity, a random effect model was employed. As demonstrated in the result of meta-analysis, LPS resulted in a decrease in the occurrence rate of complications relative to open surgery (RR = 0.83, 95% CI: 0.73 to 0.95) (Figure 5(a)) but an increase in that compared to RS (RR = 1.74, 95% CI: 1.57 to 1.92) (Figure 5(b)).

In respect of recurrence rate, 7 studies compared that in LPS and open surgery (*I*^2^ = 0.0%), and 3 studies compared that in LPS and RS (*I*^2^ = 5.3%). Because of small heterogeneity, a fixed effect model was employed. According to the result of meta-analysis, there was no notable difference in recurrence rate between LPS and open surgery (RR = 0.75, 95% CI: 0.56 to 1.01) or RS (RR = 0.97, 95% CI: 0.62 to 1.53) (Figures 6(a) and 6(b)).

#### 3.3.3. The 3-Year PFS/DFS and OS

In respect of 3-year PFS/DFS, 2 studies compared that in LPS and open surgery (*I*^2^ = 0.0%), and 3 studies compared that in LPS and RS (*I*^2^ = 90.2%). Based on the heterogeneity analysis, a fixed effect model and a random effect model were employed, respectively. The outcome of meta-analysis indicated an insignificant difference in 3-year PFS/DFS between LPS and open surgery (RR = 0.99, 95% CI: 0.90 to 1.09) or RS (RR = 1.30, 95% CI: 0.87 to 1.96) (Figures 7(a) and 7(b)).

In respect of 3-year OS, 3 studies compared that in LPS and open surgery (*I*^2^ = 0.0%), and 4 studies compared that in LPS and RS (*I*^2^ = 91.2%). Based on the results of heterogeneity analysis, a fixed effect model and a random effect model were employed, respectively. As shown in the result of meta-analysis, there was no prominent difference in 3-year OS between LPS and open surgery (RR = 0.97, 95% CI: 0.91 to 1.04) or RS (RR = 1.21, 95% CI: 0.91 to 1.60) (Figures 8(a) and 8(b)).

The article "Prognosis and Efficacy of Laparoscopic Surgery on Patients with Endometrial Carcinoma: Systematic Evaluation and Meta-Analysis" was published in 2022. Journal: Comput Math Methods Med.

## 4. Discussion

This study found that LPS did not improve the survival time of patients. A retrospective study compared the clinical effect of LPS and open surgery on the treatment of low risk EC patients (grade 1 or 2 EC and mesometrium invasion < 1/2). The result suggested that the 5-year recurrence-free survival (RFS) and OS of LPS were similar to those of open surgery [43]. Besides, another study reported the 5-year survival rate of EC patients who underwent LPS, open surgery, or RS, suggesting that there was no significant difference in 5-year DFS and OS of patients [44]. In addition, a multicenter database study verified that the long-term prognosis of MIS on treatment of high-risk EC was no worse than that of LT [45]. The above results were in agreement with the outcome of our study, which indicated that LPS did not dramatically improve the 3-year PFS/DFS and OS of patients.

Generally, LPS takes longer time on operation [36]. However, our study manifested that there was no significant difference in duration of operation between LPS and open surgery or RS. Importantly, since the duration of operation would be subjected to the skill of the operator, we could not figure out which method was the most potential to reduce the duration of operation among these surgeries. Meanwhile, the blood loss of LPS was obviously lower than that of open surgery, but it had no remarkable difference in comparison with that of RS.

The LOS of LPS was notably shorter than that of open surgery and LPS also resulted in fewer postoperative complications. However, RS was overwhelmingly better than LPS in the aspect of duration of time and postoperative complications. This study suggested that no obvious difference in recurrence rate was found between LPS and open surgery or RS.

A previous meta-analysis has proved that uterine manipulator is irrelevant to an increase in occurrence rate of positive peritoneal cytology, lymphovascular space invasion, or recurrence in EC patients [46]. Our study only investigated conventional LPS. A recent meta-analysis involved 4 RCTs that compared the clinical effect of laparoendoscopic single-site surgery (LESS) and conventional LPS on the treatment of EC patients, which suggested an insignificant difference between the two surgeries. Meanwhile, LESS only has advantage on reducing trauma [47]. Additionally, another meta-analysis that was similar to our study compared the differences between RS and LPS or open surgery. The analysis suggested that RS was characterized by less blood loss and blood transfusion, fewer postoperative complications, and less conversion to LT plus shorter LOS compared with the other two surgeries. However, RS took a longer time on operation in surgical staging of EC [48]. Interestingly, these results were consistent with the outcomes of our study. Moreover, we also analyzed the oncological outcome of EC patients.

The article "Prognosis and Efficacy of Laparoscopic Surgery on Patients with Endometrial Carcinoma: Systematic Evaluation and Meta-Analysis" was published in 2022. Journal: Comput Math Methods Med.

This study presented some advantages. Firstly, our meta-analysis involved some recent clinical trials with a vast number of samples. Furthermore, we also analyzed the survival time of patients. But few samples were involved in the analysis, which was a limitation of our study.

Inevitably, there were limitations in this study. First of all, most of the studies involved in our study were retrospective cohort studies which are inherently subjected to the risk of selection bias. Secondly, the speculation about whether various risk factors affect the prognosis of EC patients who underwent LPS is needed to be further verified. In addition, Cusimano et al. [49] performed a meta-analysis on EC patients with obesity who underwent LPS or robotic hysterectomy. The result of the analysis revealed that LPS and robotic hysterectomy had similar incidence of perioperative complications. However, robotic hysterectomy may reduce conversions due to the positional intolerance of patients suffering from morbid obesity. Finally, because of the lack of related reports on 5-year survival time of patients, we only analyzed the 3-year PFS/DFS and OS of the patients.

In summary, our study revealed that LPS was a safe and effective treatment for EC patients, which was better than open surgery. Nevertheless, LPS was at a disadvantage in the comparison with RS on duration of operation and postoperative complications. In the future, more randomized trials with complete data are needed to verify our conclusion.

## Figures and Tables

**Figure 1:** Flow chart about literature screening.

**Figure 2:** Forest plot comparing duration of operation. (a) LPS vs. open surgery; (b) LPS vs. RS.

**Figure 3:** Forest plot about the comparison on blood loss. (a) LPS vs. open surgery; (b) LPS vs. RS.

**Figure 4:** Forest plot about comparison on LOS. (a) LPS vs. open surgery; (b) LPS vs. RS.

**Figure 5:** Forest plot comparing complications. (a) LPS vs. open surgery; (b) LPS vs. RS.

**Figure 6:** Forest plot of comparison on recurrence rate. (a) LPS vs. open surgery; (b) LPS vs. RS.

**Figure 7:** Forest plot about comparison on 3-year PFS/DFS. (a) LPS vs. open surgery; (b) LPS vs. RS.

**Figure 8:** Forest plot comparing 3-year OS. (a) LPS vs. open surgery; (b) LPS vs. RS.

**Table 1:** Characteristics of literature involved.

Author	Year	Country	Center	Study design	Year of sample collection	FIGO stage	Grade	Age, mean (SD), y			BMI, mean (SD), kg/m^2^			Sample size (*n*)			Interventions			NOS
Escobar et al.	2012	USA	Multi	Retrospective cohort study	2009.4-2010.9	I-II	I-III	60.9 (12.1)	59.7 (9.2)	61.9 (11.4)	31.2 (6.7)	31.4 (6.6)	31.3 (32.0)	30	30	30	Laparoscopy	Robotic	Single-port laparoscopy	7
Wright et al.	2012	USA	Multi	Retrospective cohort study	2008.10-2010.3									1027	1437		Laparoscopy	Robotic		8
Obermair et al.	2012	Australia, New Zealand	Multi	RCT	2005.10-2010.6	IA-IVB	I-III							404	349		Laparoscopy	Open		
Goicoechea et al.	2013		Multi	Retrospective cohort study	2003.1-2010.1	I-IV	I-III	61	62		29.3	29.2		232	183		Laparoscopy	Robotic		9
Bogani et al.	2014	Italy	Single	Retrospective cohort study	2002.5-2012.10	I-IV	I-III	78	79		27	26.6		59	66		Laparoscopy	Open		9
Bogani et al.	2014	Italy	Single	Retrospective cohort study	1992.1-2013.5	I-III	I-III	83	82	84	25 (4.3)	25.4 (3.6)	28.1 (6.9)	22	25	16	Laparoscopy	Open	Vaginal surgery	8
Boosz et al.	2014		Single	Retrospective cohort study	2002.1-2009.12		I-III	63.2 (11.0)	66.7 (11.3)		29.8 (7.1)	29.7 (8.2)		107	160		Laparoscopy	Open		9
Chiou et al.	2014	China	Single	Retrospective cohort study	2005-2013	IA-IIIC		51.4 (14.2)	53.6 (11.1)	53.6 (11.3)	25.6 (5.6)	26.0 (5.2)	26.1 (5.7)	150	86	129	Laparoscopy	Robotic	Open	9
Park et al.	2015	USA	Single	Retrospective cohort study	2001.1-2012.7	IA-IVB	I-III	60	60		30.4	30.7		586	350		Laparotomy	Robotic		6
Corrado et al.	2015	Italy	Single	Retrospective cohort study	2010.8-2013.12	IA-IVB	I-III	62	63	64	29	29	28	277	72	177	Laparoscopy	Robotic	Open	6
Stefano et al.	2015	Italy	Multi	Retrospective case-control study	2000.1-2013.3	IV		62.2 (11.5)	63.2 (11.3)		27	27		764	502		Laparoscopy	Open		6
Ling-hui Chu et al.	2015	China	Single	Retrospective cohort study	2002.1-2012.6	I-III	I-III	55.3	53.4		25	25.4		70	81		Laparoscopy	Open		8
Barrie et al.	2016	USA	Single	Retrospective cohort study	2009.1-2014.1	0-IV	0-III	62	62		29.9	30.6		688	745		Laparoscopy	Robotic		9
Monterossi et al.	2016	Italian	Multi	Retrospective cohort study	2000.5-2015.6	I-II	I-III	67	69		27	27		141	142		Laparoscopy	Open		9
Beck et al.	2017	USA	Single	Retrospective cohort study	2008-2013			61 (27-90)	63 (25-96)	63 (28-94)				400	1687	1625	Laparoscopy	Robotic	Open	8
Ruan et al.	2018	Singapore	Single	Retrospective cohort study	2008-2014	I	I-III	53.0 (11.0)	55.6 (9.7)		28.1 ± 5.7	28.7 ± 6.9		145	229		Laparoscopy	Open		8
Corrado et al.	2018	Italian	Multi	Retrospective cohort study	2010-2012	I-IV	I-III	63.43	62.5		35.4 (5.8)	36.3 (6.2)		406	249		Laparoscopy	Robotic		9
Deura et al.	2018	Japan	Single	Retrospective cohort study	2005-2016	I	I-II	57	57		23.6 (15.9-48.8)	23.5 (18.0-44.6)		40	80		Laparoscopy	Open		8
Jørgensen et al.	2018	Denmark	Single	Prospective cohort study	2005.1.1-2015.6.30	I-II	I-III	67 (37-94)	67 (33-94)	68 (40-98)	178 (33.1)	361 (29.4)	245 (35.3)	569	1282	712	Laparoscopy	Robotic	Open	9
Vardar et al.	2018			Retrospective cohort study	2005.1-2016	I-IIII	I-III	35 (12.2)	61 (11.8)		35.0 (7.4)	35.8 (7.4)		286	515		Laparoscopy	Open		9
Ghazali et al.	2018	Malaysia	Single	Retrospective cohort study	2010.1-2014.12			55.62 (12.75)	57.79 (9.63)		32.57 (8.89)	29.24 (3.71)		26	14		Laparoscopy	Open		8
Dieterich et al.	2019	Germany	Single	Retrospective cohort study	2005.1-2014.12	I-III	I-III	64.00 (11.04)	66.48 (11.41)		32.49 (8.86)	33.71 (8.26)		108	242		Laparoscopy	Open		9
Papadia et al.	2019	Swiss confederation	Single	Retrospective cohort study	2001.10-2015.11	III		65 (11)	63.2 (11.2)		26.6 (7.4)	26.5 (7.2)		51	15		Laparoscopy	Open		9
Tanaka et al.	2020	Japan	Single	Retrospective cohort study	2004.1-2019.12	IA-IV	I-III	55.3 (10.6)	56.0 (10.3)		23.4 (4.4)	24.4 (4.9)		226	252		Laparoscopy	Open		8

The article "Prognosis and Efficacy of Laparoscopic Surgery on Patients with Endometrial Carcinoma: Systematic Evaluation and Meta-Analysis" was published in 2022. Journal: Comput Math Methods Med.

## Data Availability

The data used to support the findings of this study are included within the article. The data and materials in the current study are available from the corresponding author on reasonable request.
